The article "Order Management and Completion Date Prediction of Manufacturing Job-Shop Based on Deep Learning" was retracted in 2023. Reasons: unreliable results or conclusions; concerns about the data; concerns about the results or conclusions; concerns about the peer review.

# Order Management and Completion Date Prediction of Manufacturing Job-Shop Based on Deep Learning

**DOI:** 10.1155/2022/3458116

**Published:** 2022-03-16

**Authors:** Mei Wang

**Affiliations:** School of Information Science and Engineering, Shandong Agriculture and Engineering University, Jinan 250100, China

## Abstract

To cope with the volatility of customer order demand, enterprises need to formulate a reasonable production plan based on customer demand for the completion period and their current manufacturing capacity. The existing studies have not fully considered the complex processing procedures, the features of manufacturing attributes, and the repetitive orders of stable consumers. To solve these problems, this paper explores the order management and completion date prediction of manufacturing job-shop based on deep learning. Specifically, the features of manufacturing attributes were extracted and used to predict the activities and completion time of different manufacturing tasks in order management. In addition, a deep learning prediction model was constructed based on a bidirectional long short-term memory network (BiLSTM) and self-attention mechanism, which completes the order management and completion date prediction.

## 1. Introduction

With the continuous development of the market economy and the advancement of science and technology, consumers expect ordered products to be delivered within a shorter cycle [1–7]. The increasingly market-centric order production method puts forward extremely strict requirements on the corporate capacity of production and timely completion [8–10]. To cope with the volatility of customer order demand, i.e., meet consumer requirements on the quality and completion date of ordered products, enterprises need to effectively control the ordered tasks in the manufacturing job-shop and to formulate a reasonable production plan based on customer demand for the completion period and their current manufacturing capacity [11–18]. In the manufacturing industry, order management runs through the entire production cycle. The accurate prediction of the product completion period is the main factor affecting the decision of order management and control [19–22].

Chen [23] constructed a system based on the knowledge of fuzzy neural networks, aiming to improve the performance of manufacturing job-shop in predicting completion time and allocating internal delivery time. In the system, multiple experts construct their own fuzzy multiple linear regression (MLR) models and predict the job completion time/cycle. Drawing on concepts like machine learning, evolution, and metaheuristic learning, Patil [24] developed an enhanced differentiable dynamic quantization (DDQ) model based on an artificial neural network (ANN). Computational experiments show that the model outshines traditional ANN-based DDQ in the prediction of the completion date, in different job-shop environments and on different volumes of training data. To prevent overfitting from weakening the generalization ability of a single neural network, Zhu et al. [25] introduced a neural network ensemble to propose a Bagging approach based on the cluster analysis of the 0.632 prediction error and conducted a case study to illustrate the whole steps to predict the product due date by using neural network ensemble. The operation of manufacturing job-shop is difficult to manage, owing to the heterogeneity of raw materials, complex transformation process, and varied production flows. Dumetz et al. [26] provided a simulation framework enabling the comparison and evaluation of different production planning strategies and order management strategies. The framework integrates a basic enterprise resource planning (ERP) system. The user can configure the production plan and order management process and evaluate the model performance in various market environments using the discrete event simulation model. After setting up a set of candidate features, Liu et al. [27] presented a feature selection algorithm based on the self-organizing map-feature-weighted fuzzy c-means (SOM-FWFCM) algorithm. Taking the production data of a job-shop as an example, the proposed algorithm was compared with four feature selection algorithms. The comparison demonstrates the effectiveness of that algorithm.

The completion time of ordered products can be predicted well by combining data mining with the analysis of the discrete data in the manufacturing industry, which are featured by scattered distribution, large volume, and poor authenticity. However, the existing studies have not fully considered the complex processing procedures, the features of manufacturing attributes, and the repetitive orders of stable consumers. To solve these problems, this paper explores the order management and completion date prediction of manufacturing job-shop based on deep learning.  Section 2 extracts the features of manufacturing attributes, using the recursive feature elimination approach of random forest (RF), principal component analysis (PCA), and k-means clustering (KMC). Based on the extracted features, Section 3 predicts the activities and completion time of different manufacturing tasks in order management and constructs a deep learning prediction model based on bidirectional long short-term memory network (BiLSTM) and self-attention mechanism. The proposed model was proved effective through experiments.

## 2. Feature Extraction

In complex orders, the diverse products are manufactured in small batches through complicated and variable operations. As a result, it is not very desirable to predict the completion period of the products in complex orders by optimizing the processing operations of these products using heuristic algorithms. In the manufacturing job-shop, the order completion time is affected by complex, stochastic, and correlated factors. During real-world job-shop production, there is no ability to collect all the valuable and real information from the manufacturing process of ordered products. Therefore, it is particularly important to clarify the association between the information containing lots of abnormal data and the completion period of ordered products.

The completion date of ordered products is affected by the following factors: requirement on order quality, urgency of delivery, importance of consumers, profit margin of order, task volume of order, and complexity of operations. This paper proposes a hybrid algorithm for mining the factors affecting the completion period of ordered products. Firstly, the important features of manufacturing attributes were extracted by the recursive feature elimination approach of RF. Then, the linear features of manufacturing attributes were extracted through the PCA. After that, the KMC was applied to extract the nonlinear features of manufacturing attributes. Finally, the extracted important features, linear features, and nonlinear features are fully fused.

### 2.1. Extraction of Important Features

The recursive feature elimination approach of RF is detailed as follows:

*Step 1*. Perform random sampling with the replacement on the manufacturing attribute samples in the original training set *C*. Suppose there are *M* original samples, and *N* samples are selected in each sampling. Denote the *i*-th bootstrap sample set generated through multiple random repetitive sampling as *δ*_*i*_.
*Step 2.* Select the splitting feature and the splitting point with the smallest Gini index to split the decision tree (DT), and build the *i*-th nonpruned and fully grown classification and regression tree (CART) *ψ*_*i*_ based on the bootstrap sample set *δ*_*i*_. Repeat this step until all DTs are constructed.
*Step 3*. Calculate the mean square error (MSE) of the RF model. For the *i*-th DT *ψ*_*i*_, define the *M*-*N* samples not collected in the *i*-th random sampling as a set NDS_*i*_. Let *E*_*i*_^MSE^ be the MSE of DT *ψ*_*i*_, *w*_*c*_ be the true value of the test data, and *w*_*ic*_^*∗*^ be the predicted value of DT *ψ*_*i*_. Then, the MSE can be calculated by the following:
  (1) $$\begin{array}{c} E_{i}^{\text{MSE}}=\frac{\sum_{c=1}^{M-N}{\left(w_{c}-w_{ic}^{*}\right)}^{2}}{M-N}. \end{array}$$
*Step 4.* Calculate the importance score of each feature of manufacturing attributes. The importance score FR_*c*_ of feature FE_*c*_ can be calculated by the following:
  (2) $$\begin{array}{c} {\text{FR}}_{c}=\frac{1}{l}\sum_{i=1}^{l}\left({S^{\prime }}_{i}^{\text{MSE}}-S_{i}^{\text{MSE}}\right). \end{array}$$
*Step 5*. Output the feature set of manufacturing attributes corresponding to the minimum *E*_*i*_^MSE^, during the elimination of the feature with the smallest FR_*c*_.

### 2.2. Extraction of Linear Features

Let *C* = {*c*_1_, *c*_2_,…, *c*_*t*_} be the original training set composed of the column vectors of manufacturing attribute samples. In this paper, the PCA is adopted to extract the linear features from manufacturing attributes. In essence, the extraction searches for a unit projection vector *φ* that maximizes the projected variance of *c*_*i*_ on *φ*.

To eliminate the influence of the varied dimensionality between the column vectors of manufacturing attribute samples, *C* can be normalized by the following:

(3) $$\begin{array}{c} Q=\left\{q_{1},q_{2},\ldots ,q_{t}\right\}=\left\{c_{1}-e,c_{2}-e,\ldots ,c_{t}-e\right\}, \end{array}$$

where

(4) $$\begin{array}{c} e=\frac{1}{t}\sum_{i=1}^{t}c_{i}. \end{array}$$

Let Λ be the covariance matrix of sample set *Q*. The projection variance *PV*(*q*) of dataset *Q* = {*q*_1_, *q*_2_,…, *q*_*t*_} on unit vector *φ* can be calculated by the following:

(5) $$\begin{array}{c} FR\left(q\right)=\frac{1}{t}{\sum_{i=1}^{t}\left(q_{i}^{\psi }\phi \right)}^{2}=\frac{1}{t}{\sum_{i=1}^{t}\left(q_{i}^{\psi }\phi \right)}^{\psi }\left(q_{i}^{\psi }\phi \right)\\ =\frac{1}{t}\sum_{i=1}^{t}\phi^{\psi }q_{i}q_{i}^{\psi }\phi =\phi^{\psi }\left(\frac{1}{t}\sum_{i=1}^{t}q_{i}q_{i}^{\psi }\right)\phi .=\phi^{\psi }\Lambda \phi . \end{array}$$

Thus, the PCA can be converted into the following mathematical problem:

(6) $$\begin{array}{c} \left\{\begin{array}{c} \underset{\phi }{\max}\phi^{\psi }\sum \phi \\ s.t.\phi^{\psi }\phi =1 \end{array}\right). \end{array}$$

Let *μ* be the Lagrangian multiplier. Formula (6) can be solved by the Lagrangian function *U*(*φ*, *μ*):

(7) $$\begin{array}{c} U\left(\phi ,\mu \right)=\phi^{\psi }\sum \phi -\mu \phi^{\psi }\phi . \end{array}$$

Solving the partial derivative of *U*(*φ*,*μ*) for *φ*:

(8) $$\begin{array}{c} \frac{\partial U\left(\phi ,\mu \right)}{\partial \phi }=2\sum \phi -2\mu \phi =0\Rightarrow \sum \phi =\mu \phi . \end{array}$$

Combining Λ*φ* = *μφ* with formula (8):

(9) $$\begin{array}{c} FR\left(q\right)=\phi^{\psi }\left(\frac{1}{t}\sum_{i=1}^{t}q_{i}q_{i}^{\psi }\right)\phi =\phi^{\psi }\sum \phi =\mu \phi^{\psi }\phi =\mu . \end{array}$$

Formula (9) shows that the eigenvalue of the covariance matrix Λ of manufacturing attribute sample *q* is its projection variance on unit vector *φ*. The largest eigenvalue of Λ is the maximum projection variance, and the second largest eigenvalue of Λ is the next best projection variance. The rest can be obtained by analogy. The flow of the PCA is detailed as follows:

*Step 1*. Normalize the original training set *C* = {*c*_1_, *c*_2_,…, *c*_*t*_} to eliminate the influence of the varied dimensionality between the column vectors of manufacturing attribute samples. That is, ensure that the mean projection *e*′ of normalized dataset *Q* = {*q*_1_, *q*_2_,…, *q*_*t*_} on projection vector *φ* equals zero:
  (10) $$\begin{array}{c} e^{\prime }=\frac{1}{t}\sum_{i=1}^{t}q_{i}^{\psi }\phi =\left(\frac{1}{t}\sum_{i=1}^{t}q_{i}^{\psi }\right)\phi =0. \end{array}$$
*Step 2*. Compute the covariance matrix Λ of sample set *Q*:
  (11) $$\begin{array}{c} \Lambda =\frac{1}{t}\sum_{i=1}^{t}q_{i}q_{i}^{\psi }. \end{array}$$
*Step 3*. Decompose the eigenvalues of covariance matrix Λ, and sort them in descending order. Denote the ranked eigenvalues and the corresponding eigenvectors as {*ξ*_1_, *ξ*_2_,…, *ξ*_*t*_} and {*φ*_1_, *φ*_2_,…, *φ*_*t*_}, respectively.
*Step 4*. Map the eigenvectors {*φ*_1_, *φ*_2_,…, *φ*_*v*_} corresponding to the top *v* eigenvalues. Let *q*_*i*_^*N*^ be the mapped sample data. Then, the *t*-dimensional data can be mapped into *v*-dimensional data by the following:
  (12) $$\begin{array}{c} q_{i}^{\text{new}}=\left[\begin{array}{c} \phi_{1}^{\psi }q_{i}\\ \phi_{2}^{\psi }q_{i}\\ \vdots \\ \phi_{v}^{\psi }q_{i} \end{array}\right]. \end{array}$$
The cumulative contribution rate *γ* can be determined by the following:
  (13) $$\begin{array}{c} \gamma =\sqrt{\frac{\sum_{i=1}^{v}\xi_{i}^{2}}{\sum_{i=1}^{t}\xi_{i}^{2}}}. \end{array}$$

### 2.3. Extraction of Nonlinear Features

The KMC was adopted to extract the nonlinear features of manufacturing attributes. Before feature extraction, the low-dimensional data on ordered products should be mapped into high-dimensional data through the following steps:

*Step 1*. Perform feature interaction on the original training set *C* = {*c*_1_, *c*_2_,…, *c*_*t*_} and denote the resulting interactive feature set as *C'* = {*c*_0,1_, *c*_1,2_,…, *c*_*t*−1,*t*_}. Let *q*_*ij*_ be the area feature interaction result between features *q*_*i*_ and *q*_*j*_. The feature product interaction can be calculated by the following:
  (14) $$\begin{array}{c} q_{i,j}=q_{i}\times q_{j}. \end{array}$$
*Step 2*. Set the number of clusters for nonlinear manufacturing features and select an initial center randomly for each class. Find the optimal number of classes by the inflection point method for the within-cluster sum of squares, i.e., compute the within-cluster sum of squares at different *k* values. Let *SU*(*f*_1_, *f*_2_,…, *f*_*K*_) be the within-cluster sum-of-squares; *f*_*j*_ be the center of the *j*-th cluster; *q*_*i*_ be the *i*-th sample in the *j*-th cluster; *r*_*j*_ be the total number of samples in the *j*-th cluster. Then, the optimal number of clusters can be calculated by the following:
  (15) $$\begin{array}{c} SU\left(f_{1},f_{2},\ldots ,f_{K}\right)=\sum_{j=1}^{K}\sum_{i}^{r_{j}}{\left(q_{i}-f_{j}\right)}^{2}. \end{array}$$
*Step 3*. Compute the distance between each cluster center and each interactive feature in the dataset. Based on the computed results, assign the interactive feature to the right cluster. Measure that distance with cosine similarity. The cosine similarity between samples *q*_1_ and *q*_2_ can be calculated by the following:
  (16) $$\begin{array}{c} v=\frac{\sum_{i=1}^{r}q_{1i}q_{2i}}{\sqrt{\sum_{i=1}^{r}q_{1i}^{2}}\sqrt{\sum_{i=1}^{r}q_{2i}^{2}}}. \end{array}$$
*Step 4*. Update the center of each cluster based on the mean of the samples in that cluster. The partial derivative of the loss function can be calculated by the following:
  (17) $$\begin{array}{c} \frac{\partial S\;U\left(f_{1},f_{2},\ldots ,f_{h}\right)}{\partial f_{j}}=\sum_{j=1}^{h}\sum_{i}^{r_{j}}\frac{\partial {\left(q_{i}-f_{j}\right)}^{2}}{\partial f_{j}}=\sum_{i}^{r_{j}}\frac{\partial {\left(q_{i}-f_{j}\right)}^{2}}{\partial f_{j}}=\sum_{i}^{r_{j}}-2\left(q_{i}-f_{j}\right). \end{array}$$
Making formula (17) equal to zero:
  (18) $$\begin{array}{c} \sum_{i}^{r_{j}}-2\left(q_{i}-f_{j}\right)=0,\\ r_{j}f_{j}-\sum_{i}^{r_{j}}q_{i}=0\Rightarrow f_{j}=\frac{\sum_{i=1}^{r_{j}}q_{i}}{r_{j}}. \end{array}$$
Formula (18) shows that the loss is minimized, when the cluster center equals the mean of all samples in that cluster.
*Step 5.* Repeat Steps 3-4 until the termination condition is satisfied.
*Step 6*. Output the *K* cluster centers as the nonlinear features extracted from manufacturing attribute samples.

Figure 1 explains the flow of linear and nonlinear feature extractions. All completion date prediction models are verified on the test data. The above algorithm is adopted to extract the features of the factors affecting the completion date, according to the test error of each model. Then, the mean test error is computed, and the prediction model with the smallest test error is selected.

## 3. Prediction of Activities and Completion Time

Process mining of predictive order management helps job-shop managers identify abnormal, incompliant order management activities so that they could take emergency measures and crisis response measures. In the context of order management, the prediction of activities and completion time of each manufacturing task brings several advantages: effectively increasing job-shop production efficiency, significantly lowering operating costs, and accurately recognizing illegal activities.

Figure 2 presents the framework of the prediction model for order management activities and completion time. There are five layers in the framework: an input layer, an embedding layer, a BiLSTM layer, a self-attention layer, and an output layer.

The attributes in job-shop manufacturing logs should be extracted and converted into eigenvectors before being imported to the prediction model. Let *K* = {*ε*_1_, *ε*_2_, *ε*_3_,…, *ε*_*m*_} be the set of job-shop manufacturing logs, where *ε*_*i*_ = <*o*_*τ*1_, *o*_*τ*2_, *o*_*τ*3_,…, *o*_*τm*_> represents the evolutionary trajectory of the *i*-th event, with *m* = |*ε*_*i*_|. Each evolution trajectory needs to be converted into an eigenvector *a* = [*a*_1_, *a*_2_, *a*_3_,…, *a*_*GR*_], with *GR* being the number of samples. In the eigenvector *a* = [*a*_1_, *a*_2_, *a*_3_,…, *a*_*GR*_], element *a*_*i*_ is a two-dimensional eigenvector, including both the event trajectory related to completion time and the number of event-related attributes. The latter covers numerical and non-numerical attributes.

Before an eigenvector is inputted to the neural network via the embedding layer, it is necessary to linearly map the high-dimensional sparse eigenvector *a* = [*a*_1_, *a*_2_, *a*_3_,…, *a*_*GR*_]. Let *WS* be the dimensionality of the code for the mapped eigenvector. Then, the mapped low-dimensional dense eigenvector can be expressed as *o* = [*o*_1_, *o*_2_, *o*_3_,…, *o*_*τ*_], with *o*_*τ*_*∈R*^WS^. Then, we have the following:

(19) $$\begin{array}{c} \text{GR}\left(a_{1},a_{2},a_{3},\ldots ,a_{GR}|a_{i}\right)=\sum_{d=1}^{\text{GR}}\text{GR}\left(a_{d}|a_{i}\right),\\ o\left(a\right)=-\sum \sum_{i=1}^{k}\log\text{GR}\left(a_{\text{GR}}|a_{i}\right). \end{array}$$

In our embedding layer, nonnumerical attributes are encrypted by one-hot encoding. This is because one-hot encoding features high-dimensional sparsity and involves no internal association through nonlinear mapping. Every embedding vector can be updated through the network training based on the embedding layer, completing the search for similarity between different vectors in a multidimensional space [28].

The BiLSTM consists of two LSTMs with the opposite propagation directions.  Figure 3 explains the internal structure of an LSTM. As a modification of recurrent neural network (RNN), the LSTM has a strong ability of modeling time series and overcomes the memory problem and vanishing gradients of traditional RNN. The LSTM can update the hidden state YC_*τ*_, based on the input *o*_*τ*_ of the previous layer and the previous hidden state YC_*τ*−1_. Let SR_*τ*_, YW_*τ*_, and SC_*τ*_ be the input gate, forget gate, and output gate, respectively. The input gate selectively preserves the input information and updates the cell state, the forget gate selectively forgets the redundant information, and the output gate determines which cell state should be outputted. Let *ω* be the output weight; PO be the bias; JH_1_ and JH_2_ be the activation function sigmoid and the activation function tanh, respectively. Then, we have the following:

(20) $$\begin{array}{c} {\text{SR}}_{\tau }={\text{JH}}_{1}\left(\omega_{SR}*\left[{\text{YC}}_{\tau -1},o_{\tau }\right]+{\text{PO}}_{\text{SR}}\right),\\ {\text{YW}}_{\tau }={\text{JH}}_{1}\left(\omega_{g}*\left[{\text{YC}}_{\tau -1},o_{\tau }\right]+{\text{PO}}_{\text{YW}}\right),\\ {\text{GS}}_{\tau }^{\prime }={\text{JH}}_{2}\left(w_{\text{GS}}*\left[{\text{YC}}_{\tau -1},o_{\tau }\right]+{\text{PO}}_{\text{GS}}\right),\\ {\text{GS}}_{\tau }={\text{YW}}_{\tau }*{\text{GS}}_{\tau -1}+{\text{SR}}_{\tau }*{\text{GS}}_{\tau }^{\prime },\\ {\text{SC}}_{\tau }={\text{JH}}_{1}\left(\omega_{\text{SC}}*\left[{\text{YC}}_{\tau -1},o_{\tau }\right]+{\text{PO}}_{\text{SC}}\right),\\ {\text{YC}}_{\tau }={\text{SC}}_{\tau }*{\text{JH}}_{2}\left({\text{GS}}_{\tau }\right). \end{array}$$

The BiLSTM is an extension of unidirectional LSTM based on reverse time flow. Let YC′_*τ*_ and YC^″^_*τ*_ be the forward and backward order management states, respectively. Then, the current output state *YC*_*τ*_ can be updated based on YC′_*τ*_ and YC^″^_*τ*_. In addition, the one-way operation flow of the LSTM is denoted as *K*_OW_. Compared with traditional one-way LSTM, the BiLSTM learns historical and future states of order management simultaneously, and acquires highly stable and reliable feature information. Then, we have the following:

(21) $$\begin{array}{c} {{\text{YC}}^{\prime }}_{\tau }=K_{\text{OW}}^{\prime }\left({\text{YC}}_{\tau -1},o_{\tau }\right),\\ {{\text{YC}}^{\prime \prime }}_{\tau }=K_{\text{OW}}^{\prime \prime }\left({\text{YC}}_{\tau +1},o_{\tau }\right),\\ {\text{YC}}_{\tau }=\left[{{\text{YC}}^{\prime }}_{\tau },{{\text{YC}}^{\prime \prime }}_{\tau }\right]. \end{array}$$

The job-shop orders placed by a stable consumer group tend to be repetitive. In fact, repetition is an obvious feature of predicting the activities and completion time of every manufacturing task during order management. This paper adds a self-attention mechanism to the network to forecast repetitive activities.  Figure 4 explains the internal structure of the attention mechanism. The attention-based prediction model considers the weight coefficient between input eigenvectors, and the manufacturing tasks related to the current input eigenvector, without being distracted by the information weakly correlated with the current input eigenvector.

Let *x*_*τ*,*τ*′_ be the similarity matrix between hidden states YC_*τ*_ and YC′_*τ*_ at moments *τ* and *τ′*, respectively; *ω*_YW_ and *ω*_YW_′ be the weight matrices of hidden states YC_*τ*_ and YC′_*τ*_, respectively; *ω*_*x*_ be the weight matrix for nonlinear combination; PO_*x*_ and PO_YW_ be bias vectors. The vector matrix [YC_1_, YC_2_, YC_3_,…, YC_*τ*_] of the previous BiLSTM is imported to the attention layer. Then, the similarity of any feature to every neighbor can be characterized by a self-attention matrix *X*:

(22) $$\begin{array}{c} {\text{YW}}_{\tau ,\tau^{\prime }}={\text{JH}}_{2}\left(\omega_{\text{YW}}{\text{YC}}_{\tau }+\omega_{{\text{YW}}^{'}}{\text{YC}}_{\tau^{\prime }}+{\text{PO}}_{\text{YW}}\right),\\ x_{\tau ,\tau^{\prime }}=\text{JH}\left(\omega_{x}{\text{YW}}_{\tau ,\tau^{\prime }}+{\text{PO}}_{x}\right). \end{array}$$

The hidden state *τ′* of the attention at moment *τ* is the weighted sum of all hidden states YC′_*τ*_ and similarity matrix *x*_*τ*,*τ*′_ at moment *τ'*:

(23) $$\begin{array}{c} k_{\tau }=\sum_{\tau =1}^{m}x_{\tau ,\tau^{\prime }}\times YC_{\tau }. \end{array}$$

For each manufacturing task in order management, the output layer should predict both activities and completion time. The activity prediction mainly transforms order management into multiple classes of manufacturing tasks. The softmax classifier is adapted to output the predicted activities of order management and the cross-entropy loss. Let *a* be the evolution trajectory of the input manufacturing event; FS be the total classes of manufacturing tasks; *b*_*i*_ be the true label class of the *i*-th class; *g*_*i*_ (*a*) be the predicted output of the model. Then, the cross-entropy loss can be calculated by the following:

(24) $$\begin{array}{c} \text{LOSS}\left(a\right)=-\sum_{i=k}^{FS}b_{i}\log\;g_{i}\left(a\right). \end{array}$$

## 4. Experiments and Results Analysis

Taking a furniture enterprise in Foshan, southern China's Guangdong Province as an example, this paper adopts the recursive feature elimination approach of RF to extract the important features from manufacturing attributes. The lowest-ranking feature was removed, and the feature extraction error was computed. These steps were repeated until all unimportant features were eliminated.  Figure 5 reports the feature extraction errors at different numbers of residual features. It can be learned that the model was highly accurate at 5–7 residual features and relatively inaccurate at fewer than 4 residual features.

In this paper, the PCA is performed to extract the linear features of manufacturing attributes. The cumulative contribution rate was calculated under a different number of principal components (as shown in Figure 6). Referring to the cumulative contribution rates of all components, the minimum threshold was defined for the cumulative contribution rate (0.8). Hence, the top six principal components were extracted.  Table 1 shows the linear features extracted from the manufacturing attributes in view of the factors affecting the order completion period.

Next, the KMC was called to extract the nonlinear features of manufacturing attributes. The optimal number of clusters was determined as 15 by the inflection point and the within-cluster sum-of-square. After that, a cluster analysis was carried out on interactive features.  Table 2 shows the nonlinear features extracted by KMC from manufacturing attributes.

The prediction performance of our model on manufacturing activities and completion time for ordered products was evaluated through experiments on a self-designed manufacturing attribute sample set. The sample set was divided into a training set and a test set by the ratio of 3 : 1. One-eighth of the training set was organized as a verification set.  Figure 7 shows the training loss curve of our prediction model for the completion period. The curve demonstrates the convergence ability of our model.

Our prediction model was applied to predict the manufacturing activities and completion time on samples from different sources (as shown in Table 3). The prediction accuracy and error of our model were compared with those of stacked autoencoder and 1DCNN. From the manufacturing sample sets from different job-shops, the trajectories of manufacturing events with repeatable features involving orders from stable consumers were screened. In addition, our model was compared separately with the stacked autoencoder.  Figure 8 compares their prediction accuracies of repetitive activities on samples from different sources. Facing samples from different sources, our model was far more accurate in predicting repetitive activities than the stacked autoencoder. Of course, our model performance is slightly insufficient on the self-designed dataset: the learning ability was not fully exerted, and the obvious features of manufacturing attributes were not ideally extracted. The reason is that the manufacturing events in the job-shops are executed manually, which brings certain stochastic and changeable factors. In spite of that, the experimental results demonstrate that our model is feasible to predict the completion period of orders with repeatable features laid by stable consumers.

Next, our prediction model for the completion period of ordered products, which was constructed based on the features extracted from manufacturing attributes, was compared with machine learning through experiments.  Table 4 shows the experimental results of the two prediction models on the test data. The results fully demonstrate the effectiveness of our model.  Figure 9 compares the predicted value of our model with the true value. The small error between the two values visually demonstrates the superiority of our model in prediction.

## 5. Conclusions

Based on deep learning, this paper explores the order management and completion date prediction of manufacturing job-shop. Firstly, the important features, linear features, and nonlinear features were extracted from manufacturing attributes. Next, a deep learning prediction model was constructed based on BiLSTM and the self-attention mechanism. Based on the extracted features, the manufacturing task activities and their completion time were forecasted by the proposed model. Through experiments, the relevant features were extracted from manufacturing attributes by the recursive feature elimination approach of RF, PCA, and KMC. The training loss curve of the completion period prediction model was plotted, revealing the convergence ability of the model. In addition, our prediction model was applied to predict manufacturing activities and completion time on samples from different sources. The prediction error and accuracy were summarized. Furthermore, the experimental results of our model were compared with those of stacked autoencoder and 1DCNN. The comparison visually demonstrates the superior prediction effect of our model.

## Figures and Tables

**Figure 1:** Flow of linear and nonlinear feature extractions. (a) Linear feature extraction; (b) nonlinear feature extraction.

**Figure 2:** Prediction model for order management activities and completion time.

**Figure 3:** Internal structure of an LSTM.

**Figure 4:** Internal structure of attention mechanism.

**Figure 5:** Feature extraction errors vs. number of residual features.

**Figure 6:** Cumulative contribution rate vs. number of principal components.

**Figure 7:** Training loss curve of completion period prediction model.

**Figure 8:** Prediction accuracies of repetitive activities on data from different sources.

**Figure 9:** Predicted value vs. true value.

**Table 1:** Results of linear feature extraction.

Serial number	1	2	3	4	5	6	7	…	20
First principal component	0.8605	−0.9658	0.6122	0.9354	0.3251	0.7523	−0.8695	…	1.1352
Second principal component	0.7258	1.5384	2.0314	0.3528	−1.6583	−2.2587	−2.8391	…	1.0038
Third principal component	0.0358	−0.3623	0.5682	−0.3529	−0.0595	−1.1536	0.1853	…	2.3844
Fourth principal component	2.1059	−1.0568	0.2685	1.7682	1.1582	1.6569	0.3587	…	0.2859
Fifth principal component	−0.2341	−0.9659	0.5623	1.7862	1.1456	1.6852	0.3865	…	0.2752
Sixth principal component	−0.2694	−0.2381	0.6852	1.0586	0.6387	−0.5283	−0.9381	…	−0.8375

**Table 2:** Results of nonlinear feature extraction.

Serial number	1	2	3	4	5	6	7	8	…	20
Feature-1	0.3652	0.3424	0.3976	0.0531	0.0283	0.1385	0.0869	0.1859	…	0.2541
Feature-2	0.6831	0.3157	0.3867	0.2735	0.0586	0.0853	0.1867	0.1527	…	0.3856
Feature-3	0.5672	0.0725	0.5282	0.4685	0.3652	0.8594	0.0685	0.0267	…	0.8659
Feature-4	0.8693	0.9658	0.3254	0.0823	0.0428	0.0725	0.2843	0.3048	…	0.5428
Feature-5	0.2864	0.6859	0.4857	0.3257	0.2527	0.2576	0.0865	0.2375	…	0.1586
Feature-6	0.4586	0.0527	0.2586	0.5861	0.3458	0.3528	0.3157	0.2542	…	0.3425

**Table 3:** Experimental results of different models.

Source	Job-shop 1			Job-shop 2		
Model type	Our model	Stacked autoencoder	1DCNN	Our model	Stacked autoencoder	1DCNN
Prediction accuracy of manufacturing activities	79.15	74.52	71.51	77.35	76.26	71.38
Prediction error of completion time	1.65	2.41	—	1.56	1.61	—

Note: 1DCNN is short for the one-dimensional convolutional neural network.

**Table 4:** Experimental results of the two prediction models.

Model number			1	2	3	4	5	6	7	8
Feature extraction method			Machine learning	Machine learning	Machine learning	Our model	Our model	Our model	Machine learning	Our model
Test samples	30.25	Results on completion period prediction model	32.86	29.65	30159	30.59	30.58	30.84	31.86	30.86
	39.68		34.68	3567	38.67	39.75	39.64	39.05	40.56	39.57
	35.86		36.28	34.58	36.24	35.67	35.28	35.58	34.28	35.54
	40.58		41.53	39.67	41.25	40.58	40.58	40.91	42.38	40.57
	38.53		37.86	36.82	37.58	38.48	38.82	38.81	37.12	38.58

## Data Availability

The data used to support the findings of this study are available from the author upon request.
